# The Significance of Intracranial Pressure Monitoring for Reducing Mortality in Patients with Traumatic Brain Injury: A Systematic Review and Meta-Analysis

**DOI:** 10.1155/2022/1956908

**Published:** 2022-10-08

**Authors:** Nianchen Han, Fan Yang, Xianghe Zhang

**Affiliations:** Department of Neurosurgery, The First Hospital of China Medical University, Shenyang, 110001 Liaoning, China

## Abstract

**Background:**

Despite guidelines provided by the Brain Trauma Foundation (BTF) for treating patients with TBI, including advice to monitor intracranial pressure (ICP), the clinical application of ICP monitoring is far from universal. This laxity has been attributed to the relationship between mortality in TBI patients and ICP monitoring.

**Objective:**

This systematic review and meta-analysis was aimed at determining the effect of intracranial pressure (ICP) monitoring on the mortality of patients with traumatic brain injury (TBI).

**Method:**

A systematic search for articles was conducted on PubMed, Scopus, Cochrane Central Register of Control Trials (CENTRAL), and APA PsycNet for articles published from 1 January 2000 to 1 August 2022. Manager 5.4 was used to carry out statistical analysis.

**Results:**

Article search yielded 1421 articles, but only 23 cohort studies were included in the systematic review and meta-analysis. The total number of study participants is 80,058. Seventeen studies reported unadjusted odds ratios (OR), and only 8 reported the adjusted odds ratio (OR). Nine out of seventeen studies reported an unadjusted OR of less than 1, and five out of eight studies reported an adjusted OR of less than 1. From this paper's analysis, the OR for in-hospital mortality was 1.01 [95% CI, 0.80, 1.28], with a *p* value of 0.92. OR for ICU mortality was 0.84 [95% CI, 0.52, 1.35], with a *p* value of 0.47.

**Conclusion:**

But due to conflicting results, as evident above, it is unsatisfyingly challenging to draw any substantial conclusions from them. This paper thus calls for more research on this particular paper.

## 1. Introduction

As defined by the Center for Disease Control and Prevention (CDC), TBI is a disruption in the brain's normal function that can be brought on by a blow, bump, or jolt to the head or by a penetrating head injury [1, 2]. On severity, TBI can be categorized into mild traumatic brain injury (mTBI/concussion) and severe traumatic brain damage [3]. The effects of suffering from TBI may be physical, cognitive, social, emotional, or behavioral, and the results range from complete recovery to death or permanent disability [4, 5]). As stated by Yuan, Wu, Sun, et al., [6], some of the most common causes of TBI are vehicle accidents, collisions, and falling. These are all incidences involving changes in the intracranial pressure and blood flow to the brain [4].

Due to how commonplace the events that cause TBI are, it has recently become a usual cause for emergency response and medical intervention. According to statistics in the United States [2, 7, 8], 223,000 people were hospitalized in 2019 due to TBI, and the recorded death rate for the year 2022 is 176 people per day. The rate is cumulatively due to TBI and TBI-related injuries [2]. In a research paper by Langlois et al. [9], TBI was responsible for about 50,000 annual deaths and 235,000 hospital admissions in the United States for the year 2018. Also, according to Korley et al. [10], 52% of all emergency evaluations each year in the US were due to TBI. Emergency room visits, hospital admissions, and TBI-related deaths have a corresponding incidence of 78.2%, 18.5%, and 3.3% [11].

These statistics clearly indicate the global burden posed on humankind by this ailment, and despite significant advancements in neurocritical care, since its inception in the 1950s, TBI is still a high-rate cause of death [5, 12, 13].

TBI, in general, maybe a common occurrence, but TBI injuries are different in terms of severity [14]. Most TBI cases are mild, and according to Rosso et al. [15], severe TBI only occurs in 5% of TBI patients. TBI in typical cases requires rest and no other specific treatment. On the other hand, severe cases of TBI may require fixing skull fractures or removing blood clots or pools and relieving intracranial pressure inside the skull [13, 14]. According to [16], ICP levels between 10 and 20 mmHg in adults, 3 and 7 mmHg in children, and 1.5 and 6 mmHg in newborns are believed to be suitable for the brain's proper operation. Noticeable effects of elevated intracranial pressure are problems in balance, severe headaches, dizziness or vomiting, disorientation, poor coordination, and vision problems [17–19]. The process of monitoring and keeping ICP constrained within set levels is referred to as intracranial pressure (ICP) monitoring [13, 16].

Rodríguez-Boto et al. [16] state that intracranial pressure monitoring is done by placing a detection probe within the skull to measure the pressure of the contents of the cranial cavity on its walls; the corresponding waveform of intracranial pressure is then transmitted to a workstation [20]. Continuous intracranial pressure monitoring can identify abnormal shifts in intracranial pressure as soon as possible and quick and efficient treatment can stop the development of brain herniation and stop the situation or injury from worsening [21].

Guidelines by the Brain Trauma Foundation for managing patients with severe traumatic brain injury include the advice to monitor intracranial pressure (ICP) [22, 23]. Even though most scientific organizations, including BTF, have endorsed the use of ICP monitoring, its application is far from universal. For instance, ICP monitoring was employed by 63% of Canadian neurosurgeons in more than 75% of recommended cases, 15% in 25–50%, and 7% in less than 25%, according to a study of Canadian neurosurgeons [24].

One reason for this study report may be because the advantages of ICP monitoring have frequently been called into question, and some of its advantages have not been agreed upon [25]. Two surveys done by Cremer et al. [26] and Mauritz et al. [27] concluded that ICP monitoring had no clinical advantages. In contrast to these results, retrospective investigations by Bulger et al. [28] and Lane et al. [5] showed that patients who underwent ICP monitoring had better functional, survival, and mortality outcomes. With such a scope of studies being in disagreement, it becomes a dilemma to establish if ICP monitoring is advantageous or not, particularly concerning patient mortality.

## 2. Study Objective and Research Question

The Brain Trauma Foundation (BTF) guidelines recommend ICP monitoring for all patients who have experienced severe TBI (Glasgow Coma Scale (GCS) score < 9, with a CT scan revealing intracranial pathology (level II recommendation)) [21, 23, 29–31]. Despite the existing guidelines, some studies have reported on the laxity of ICP monitoring for TBI patients. Some of the reasons cited by researchers is that previous studies have not come to a definite conclusion if ICP monitoring has benefits for the patients or not.

Due to the inconclusive nature of recent research on the particular topic, this systematic review and meta-analysis was carried out to determine the effect of intracranial pressure monitoring on the mortality rate for patients with traumatic brain injury.

### 2.1. Research Question

What is the impact of intracranial pressure monitoring on the mortality rate of patients with traumatic brain injury?

## 3. Research Methods

### 3.1. Search Strategy

This systematic review and meta-analysis was carried out following guidelines outlined in the Preferred Reporting Items for Systematic Review and Meta-Analysis (PRISMA) statement [32] A systematic search for articles was conducted on PubMed/MEDLINE, Scopus, Cochrane Central Register of Control Trials (CENTRAL), and APA PsycNet for articles published from 1 January 2000 to 1 August 2022. The reference lists of the identified articles were further scanned to identify additional studies. Since only electronic databases were searched, grey literature was not taken into consideration. The purpose of the NICE guidelines is to encompass as wide a range of presentations as possible and provide safe advice to those who may have little or no specialist knowledge. This includes all head injury rather than specifically traumatic brain injury (TBI) [33–35]. It makes recommendations about time to CT and transfer of severe TBI to specialist care, and we have presented the relevant adherence figures within this report. To conduct e-databases search, a search string was developed for PubMed and then slightly adjusted for use in the other databases. The search strings used in each of the databases mentioned above are provided in Table 1.

### 3.2. Inclusion Criteria

The studies selected for this review had to be written in English and published between 1 January 2000 and 1 August 2022. The duration of carrying out the study did not matter. The characteristics based on study design, study population, publication date, and study objective were determinants if a paper was to be included in this systematic review and meta-analysis. For a research paper to be eligible, it had to meet the following criteria.

1. Original publications, which may include randomized clinical trials (also known as RCTs), retrospective cohort studies, prospective cohort studies, and case-control studies
2. Research that used a comparative approach to its design. In this study, individuals with TBI who were monitored with ICP were contrasted with patients who did not undergo ICP monitoring. Studies that did not include two clearly defined groups—an intervention group (including ICP monitoring) and a control group (with non-ICP monitoring)—were not considered for inclusion in the study or analysis
3. Articles in which the patient death rate was one of the outcomes that was evaluated as a result of the ICP monitoring intervention

### 3.3. Exclusion Criteria

All nonoriginal articles like systematic reviews, literature reviews, comments on published papers, letters to editors, and conference papers were excluded. Studies that did not report on the effect of ICP monitoring on mortality rate, non-full-text articles, and non-peer-reviewed journal articles were also excluded.

## 4. Review Methods

### 4.1. Methodological Quality Assessment

The quality appraisal criteria used in this systematic review is a modification of the STROBE initiative assessment criteria developed by von Elm et al., [35]. The original criteria was earlier used by Yuan, Wu, Sun, et al., [6]. The STROBE criteria was initially developed for cohort, case-control, and cross-sectional studies. Hence, it had to be slightly modified to assess the quality of RCTs. The criteria items and interpretation are shown in Table 2.

### 4.2. Data Extraction

After study selection and assessment of methodological quality, the next process was data extraction. Data from the eligible studies, we entered into two already prepared excel spreadsheets. The first table details how the study was carried out. The extracted data fields are author, publication year, study design, study region, number of study patients, and inclusion criteria employed in the study. The second data sheet contained data on the outcome (in-hospital and ICU mortality). Data fields in the second table are study author and year, type of mortality measure (in-hospital or ICU mortality), total study population, number of patients in the ICP and non-ICP groups, number of death cases in ICP and non-ICP groups, unadjusted and adjusted OR reported using a 95% confidence interval (CI), and confounding factors.

### 4.3. Assessment of Heterogeneity

Heterogeneity across included studies was assessed using *p* value and *I*^2^ statistics. A *p* value of less than 0.10 was considered evidence of heterogeneity. An *I*^2^ index between 50% and 70% was regarded as substantial heterogeneity, while the *I*^2^ value of more than 70% was considered ultimate proof of study heterogeneity.

### 4.4. Statistical Analysis

The tool used for statistical analysis to compute OR and generate forest and funnel plots is Review Manager 5.4. The measure of effect used was the odds ratio (OR), and it was calculated using a random effects model. A *p* value of < 0.05 was adopted as the significance threshold.

## 5. Results

### 5.1. Search Results

The search of articles in e-databases yielded 1,300 articles: three hundred and twenty-five articles from PubMed, 861 from Scopus, 88 clinical trials from CENTRAL, and 26 articles from APA PsycNet. Additional 121 articles were identified from screening reference lists, making the total number 1421. The abstracts and titles of 921 articles were screened, and 723 of them were excluded. The remaining 198 articles were read in full; only 23 met the criteria for inclusion in this systematic review and meta-analysis. The data selection process is provided in the flow graph shown in Figures 1–3 and Table 3.

### 5.2. Results of Quality Appraisal

From Table 3, we could found the results of quality appraisal.

### 5.3. Data Extraction Results

From Table 4, we could find the data extraction results.

### 5.4. Results of Individual Studies: Summary

This systematic review and meta-analysis included 23 cohort studies: eighteen retrospective cohort studies, four prospective cohort studies, and one observational cohort study. The total number of study participants is 80,058. Al Saiegh et al. [37] had the highest study population of 36,929, and Gao et al. [41] had the lowest study population of 36 patients. ICP monitoring was done in 17,651 patients compared to 62,347 patients who did not receive any ICP monitors. Only 17 studies reported unadjusted odds ratios (OR), and only 8 reported the adjusted odds ratio (OR). Predicted mortality is 36%, and the actual value is 40% (38.7–42.1% 95% CI) (Table 5).

### 5.5. Reported Odds Ratio

The results for unadjusted OR for in-hospital mortality varied substantially across studies. Nine studies (Ahl et al. [36], Barami et al. [14], Delaplain et al. [4], Gao et al. [41], Haddad et al. [42], Lane et al. [5], Mauritz et al. [13], Piccinini et al. [44], and Shafi et al. [48]) reported an odds ratio > 1, all concluding that ICP monitoring had a negative impact on the mortality of patients with TBI. On the other hand, Alali et al. [38], Farahvar et al. [40], MacLaughlin et al. [43], Rønning et al. [47], Talving et al. [49], Thompson et al. [50], and Zeng et al. [53] reported an OR of less than 1, concluding that ICP monitoring was effective in reducing the death rate of TBI patients.

When the adjusted ORs for in-hospital mortality were looked at, Al Saiegh et al. [37], Haddad et al. [42], and Shafi et al. [48] had reported an OR greater than 1. On the hand, Alali et al. [38], Farahvar et al. [40], Rønning et al. [47], Talving et al. [49], and Thompson et al. [50] reported an OR of less than 1.

For unadjusted OR rates for ICU mortality, Haddad et al. [42] and Mauritz et al. [13] reported odds ratios of 1.19 (95% CI, 0.51–2) and 1.04 (0.87–1.25). Both reported that ICP monitoring negatively impacted the mortality of TBI patients in the ICU. Mauritz et al. [27] reported an OR of 0.85 (95% CI, 0.84–0.87), noting a 29.88% death rate in the ICP group compared to the 33.11% in the non-ICP group.

The most common confounding factors reported by studies are age, sex, mechanism of injury, head abbreviated injury scale (AIS), CT scan findings, and injury severity measured using injury severity score (ISS).

### 5.6. ICP Monitoring vs. Non-ICP Monitoring: Meta-Analysis Results

This meta-analysis was conducted using two different outcomes: in-hospital mortality and ICU mortality. Quantitative data on study outcome among studies was presented in terms of death cases in each group. The groups were those who had received ICP monitoring vs. those who had not received ICP monitoring. The unadjusted and adjusted odds ratios were presented in some but not all the studies. The way data was presented made it possible to carry out a meta-analysis for the dichotomous data type by looking at the proportion of death cases in total cases within each group.

### 5.7. In-Hospital Mortality

Quantitative data used in this analysis is from Ahl et al. [36], Al Saiegh et al. [37], Alali et al. [38], Barami et al. [14], Dawes et al. [39], Delaplain et al. [4], Farahvar et al. [40], Gao et al. [41], Haddad et al. [42], Lane et al. [5], MacLaughlin et al. [43], Mauritz et al. [13], Piccinini et al. [44], Rahmanian et al. [45], Rønning et al. [47], Shafi et al. [48], Talving et al. [49], Thompson et al. [50], You et al. [51], Yuan, Wu, Yu, et al., [52], and Zeng et al. [53]. In assessing the outcome of in-hospital mortality, the total number of people included was 77,399: 16,169 in the ICP group and 61,230 in the non-ICP group. The death rates were 29.36% in the ICP group vs. 26.73% in the non-ICP group.

A random effects model was used. The calculated odds ratio (OR) was 1.01 [95% CI, 0.80, 1.28], with a *p* value of 0. The included studies had high heterogeneity of *p* < 0.00001 and *I*^2^ = 95%. The overall results showed that ICP monitoring tends to have a negative effect on the in-hospital mortality rate compared to when ICP monitoring is not used. However, these results are statistically insignificant.

Due to different publication dates, it was possible to do a subgroup analysis. The studies were split into three groups: 2000-2010, 2011-2015, and 2016-present. The subgroup results differed broadly, with a Chi^2^ = 9.19 and df = 2 (*p* = 0.01). The computed OR values for the subgroups are provided in Table 6.

The subgroup analysis showed that ICP monitoring positively impacted the reduction of mortality rates for the period between 2011 and 2015. Only these results were statistically significant, among all three, with a *p* value below the significance threshold. Also, these results had the highest computational weight. The other two subgroups, for studies conducted from 2000 to 2010 and 2016 to 2022, showed that ICP monitoring negatively impacted mortality (Table 6 and Figure 4).

### 5.8. ICU Mortality

Quantitative data used in this analysis is from Haddad et al. [42], Mauritz et al. [27], Mauritz et al. [13], and Robba et al. [46]. In assessing the outcome of ICU mortality, the total number of people included was 5,125, 2,665 in the ICP group and 2,460 in the non-ICP group. The death rates were 36.06% in the ICP group vs. 36.46% in the non-ICP group (Figures 4 and 5.

A random effects model was used, and the calculated odds ratio (OR) was 0.84 [95% CI, 0.52, 1.35], with a *p* value of 0.4. The included studies had high heterogeneity (*p* < 0.00001 and *I*^2^ = 91%). The overall results showed that ICP monitoring tends to have a positive impact on reducing the mortality rate in the ICU compared to when ICP monitoring is not used. However, these results are statistically insignificant since the *p* value is above the adopted significance threshold (Figures 6 and 7.

## 6. Discussion

It is clear that one of the primary reasons for the failure to adopt intracranial pressure (ICP) monitoring for TBI patients is a lack of scientific data that is securely grounded. This mistrust is based on the fact that there are not enough data available to definitively justify the use of ICP monitoring for TBI patients. Because of this, a comprehensive and definitive response to this knowledge gap was sought out via the use of a meta-analysis and a systematic review. According to the findings, ICP monitoring has a tendency to have a detrimental effect on the overall mortality rate in hospitals, whereas it has a beneficial effect on the mortality rate in intensive care units. Both of these findings are statistically insignificant, and as a consequence, it is very challenging to draw any meaningful inferences from them. This is an unsatisfactorily frustrating situation.

The adjusted odds ratios (OR) from included studies were also examined and compared to the analysis results in this paper. The adjusted ORs for five of the eight included papers were less than 1. These five studies reported that ICP monitoring had an effect on reducing the mortality rate for TBI patients. When comparing these results to those in this meta-analysis, it is essential to remember that this paper's analysis results are not statistically significant. It might be valid to assume that there is a proven benefit to using ICP monitoring for patients with TBI.

It becomes harder to reach a conclusion when the results for the in-hospital mortality subgroups are looked at. The only statistically significant results are from 2011 through 2015, OR = 0.71 [95% CI, 0.56 - 0.91]. These results show that ICP monitoring has a positive effect on reducing in-hospital mortality, compared to the other two subgroups' results which contradict these results but are statistically insignificant. Considering a 2/3 majority proportion, it may be prudent (though not scientifically accurate), to say that cases of in-hospital mortality increase due to the use of ICP monitoring.

Some of the most noticeable limitations encountered in carrying out this meta-analysis are the lack of different types of study design. All 23 included studies were of a cohort design, some of an observational nature, and some of retrospective nature. Another limitation may be the study population size; the study population was above 80,000, but some included studies had a number as low as 36 people [41]. It should also be noted that the meta-analysis done in this paper was based on percentage occurrences (deaths/total patients). No analysis was done to mitigate any potential effects arising from confounding factors. When interpreting the meta-analysis results, it will be useful to take this into consideration. On the other hand, the association of commonly used antibiotics with mortality and infection is also of concern [18, 19, 54].

## 7. Conclusion

In accordance with the research question formulated in this research paper, a systematic review and meta-analysis was carried out. The results from this research paper can be summarized as follows:

- Based on study data, 9 out of 17 studies reported an unadjusted OR of less than 1
- Based on study data, 5 out of 8 studies reported an adjusted OR of less than 1
- Based on this paper's meta-analysis, the OR for in-hospital mortality is 1.01 [95% CI, 0.80, 1.28], with a *p* value of 0. The OR for ICU mortality was 0.84 [95% CI, 0.52, 1.35], with a *p* value of 0. Both results are statistically insignificant [6, 52, 55]

The contradiction between subgroups in in-hospital mortality and ICU mortality leads this research paper to make the conclusion that ICP monitoring produces lower death rates when used in intensive care units (ICU). Due to the conflicting findings in (ii) and (iii), it can be assumed that the outcome of mortality due to ICP monitoring may be prone to effects from other confounding factors than earlier established. This paper calls for further research into this topic.

## Figures and Tables

**Figure 1:** Admission emergency evaluation.

**Figure 2:** PRISMA flowchart.

**Figure 3:** Emergency evaluation associations with mortality.

**Figure 4:** Forest plot of comparison: ICP vs. non-ICP.

**Figure 5:** Funnel plot of comparison: ICP vs. non-ICP.

**Figure 6:** Forest plot of comparison: ICP vs. non-ICP.

**Figure 7:** Funnel plot of comparison: ICP vs. non-ICP.

**Table 1:** Search strings.

Database	Search string
PubMed/APA PsycNet	(“intracranial pressure monitoring” OR “ICP monitor”) AND (TBI OR “traumatic brain injury” OR “craniocerebral trauma” OR “brain trauma” OR “intracranial pressure”) AND (mortality OR death)
Scopus	TITLE-ABS-KEY ((“intracranial pressure monitoring” OR “ICP monitor”) AND (tbi OR “traumatic brain injury” OR “craniocerebral trauma” OR “brain trauma” OR “intracranial pressure”) AND (mortality OR death)) AND PUBYEAR >1999 AND PUBYEAR >1999
CENTRAL	(“intracranial pressure monitoring” OR “ICP monitor”) AND (TBI OR “traumatic brain injury” OR “craniocerebral trauma” OR “brain trauma” OR “intracranial pressure”) AND (mortality OR death) in Title Abstract Keyword - with Cochrane Library publication date Between Jan 2000 and Jan 2022 (Word variations have been searched)

Note: a date filter from 2000 to 2022 was applied when searching the databases.

**Table 2:** Quality assessment criteria.

Quality criteria	Interpretation
Abstract	The abstract is well summarized and informative of what was done in the study
Objective	The study objective is clearly stated and leaves no room for misinterpretation
Study design and setting	There is a clear elaboration of how the study was done, including location, dates, exposures, and intervention
Study variables	All outcomes, exposures, factors, and confounding factors are well identified and clearly defined
Statistical methods	There is a clear definition of how quantitative data was handled and the tools used (if any)
Results	The provided study results should be relevant to the research question
Limitations	The authors established any study limitations encountered

**Table 3:** Quality appraisal.

Study	Assessment item						
	Abstract	Objective	Study design	Study variables	Statistical methods	Results	Limitations
Ahl et al. [36]	●	●	●	●	●	●	●
Al Saiegh et al. [37]	●	●	●	●	●	●	●
Alali et al. [38]	●	●	●	◌	●	●	◌
Barami et al. [14]	●	●	●	●	●	●	◌
Dawes et al. [39]	●	●	●	●	●	●	●
Delaplain et al. [4]	●	●	◌	◌	●	●	◌
Farahvar et al. [40]	●	●	●	●	●	●	●
Gao et al. [41]	●	●	●	◌	●	●	●
Haddad et al. [42]	●	●	●	●	●	●	●
Lane et al. [5]	●	●	●	●	●	●	●
MacLaughlin et al. [43]	●	●	●	◌	●	●	◌
Mauritz et al. [27]	●	●	◌	●	●	●	●
Mauritz et al. [13]	●	●	●	●	●	●	●
Piccinini et al. [44]	●	●	●	●	●	●	◌
Rahmanian et al. [45]	●	●	●	●	●	●	●
Robba et al. [46]	●	●	●	●	●	●	●
Rønning et al. [47]	◌	●	●	●	●	●	●
Shafi et al. [48]	●	●	●	●	●	●	●
Talving et al. [49]	●	●	●	◌	●	●	●
Thompson et al. [50]	◌	●	●	●	●	●	●
You et al. [51]	●	●	●	◌	●	●	◌
Yuan, Wu, Yu, et al., [52]	●	●	●	●	●	●	◌
Zeng et al. [53]	●	●	●	●	●	●	●

Note: full circle (●) means the assessment item is clearly stated, and an empty circle (○) means that the item is not stated, while a dotted circle (◌) means that the item is unclearly stated.

**Table 4:** Study demographics.

Author and year	Study design	Study region	No. of patients	Inclusion criteria
Ahl et al. [36]	Retrospective observational cohort study	USA	1154	Abbreviated injury scale (AIS) head of ≥3 and Glasgow coma scale (GCS) of ≤8
Al Saiegh et al. [37]	Retrospective observational cohort study	USA	36929	GCS < 9
Alali et al. [38]	Retrospective cohort study	US, Canada	10628	AIS head > 3 and GCS < 9 satisfy BTF criteria for ICP monitoring
Barami et al. [14]	Retrospective cohort study	US	199	GCS < 9, age ≥ 18 years
Dawes et al. [39]	Retrospective cohort study	US	822	Blunt injury, GCS ≤ 8, and abnormal intracranial findings on head computed tomography (CT)
Delaplain et al. [4]	Retrospective cohort study	US	3808	Age ≤ 16 years, GCS ≤ 8
Farahvar et al. [40]	Retrospective cohort study	USA	1307	GCS < 9
Gao et al. [41]	Retrospective cohort study	China	36	AIS head > 3 and GCS < 9 satisfy BTF criteria for ICP monitoring
Haddad et al. [42]	Retrospective cohort study	Saudi Arabia	477	GCS < 9
Lane et al. [5]	Retrospective cohort study	Canada	5487	AIS head > 3
MacLaughlin et al. [43]	Retrospective observational cohort study	USA	123	GCS ≤ 8 with intracranial hemorrhage
Mauritz et al. [27]	Retrospective observational cohort study	Austria	415	GCS < 9
Mauritz et al. [13]	Observational cohort study	Austria	1856	GCS < 9
Piccinini et al. [44]	Retrospective cohort study	USA	4880	AIS > 3, GCS < 9
Rahmanian et al. [45]	Retrospective cohort study	Iran	120	Age ≥ 18 years, GCS ≤ 8
Robba et al. [46]	Prospective observational cohort study	International (42 countries)	2367	Age ≥ 18 years, GCS eye response score of 1 (no eye opening), and GCS motor response score ≤ 5 (not obeying commands)
Rønning et al. [47]	Retrospective observational cohort study	Norway	1327	Age ≥ 12 years, GCS < 9, and AIS scores ≥ 2
Shafi et al. [48]	Retrospective cohort study	USA	1646	GCS < 9
Talving et al. [49]	Prospective cohort study	USA	216	AIS head > 3 and GCS < 9 satisfy BTF criteria for ICP monitoring
Thompson et al. [50]	Retrospective observational cohort	USA	4251	Age 24–65 yrs, ICD-9 code
You et al. [51]	Observational, prospective cohort study	China	166	Age ≥ 65 years, GCS < 9
Yuan, Wu, Yu, et al., [52]	Retrospective observational multicenter study	China	1676	Age > 14 years, GCS ≤ 12
Zeng et al. [53]	Prospective cohort study	China	168	GCS < 12

**Table 5:** Partial clinical data statistics.

Total	69.299 (100.0)	2240 (3.2)	33,327 (100.0)
Male	31.601 (45.6)	1090 (3.4)	15,297 (45.9)
Age (y) (mean (SD))	70.7 (11.7)		70.4 (11.9)
M54	6934 (10.0)	67 (1.0)	3697 (11.1)
55-64	13.461 (19.4)	259 (1.9)	6613 (19.8)
65-74	19,765 (28.5)	618 (3.1)	9422 (28.3)
75-84	21.609 (31.2)	911 (4.2)	9776 (29.3)
285	7530 (10.9)	385 (5.1)	3819 (11.5)
Laboratory results			
Blood urea nitrogen (>40 mg/dL)	4474 (6.5)	477 (10.7)	2108 (6.3)
Blood urea nitrogen (31-40 mg/dL)	5097 (7.4)	312 (6.1)	2485 (7.5)
Blood urea nitrogen (26-30 mg/dL)	5329 (7.7)	254 (4.8)	2591 (7.8)
pH arterial (§7.30)	5966 (8.6)	655 (11.0)	2917 (8.8)
Albumin (2.4 g/dL)	948 (1.4)	128 (13.5)	542 (1.6)
Albumin (2.5-3.0 g/dL)	4315 (6.2)	295 (6.8)	2274 (6.8)
White blood cell (>19.8 k/mm^3^)	3469 (5.0)	283 (8.2)	1576 (4.7)
White blood cell (14.2-19.8 k/mm^3^)	8587 (12.4)	409 (4.8)	4082 (12.2)
White blood cell (10.9-14.1 k/mm^3^)	13,031 (18.8)	457 (3.5)	6414 (19.2)
Creatine phosphokinase (M35 or >500 U/L)	8670 (12.5)	469 (5.4)	4280 (12.8)
PO (50 or >140 mm Hg)	5047 (7.3)	437 (8.7)	2305 (6.9)
Sodium (£135 or >145 mEq/L)	17.115 (24.7)	729 (4.3)	8067 (24.2)
Hemoglobin (£11 or>18 g/dL)	10,700 (15.4)	649 (6.1)	5554 (16.7)
Potassium (>4.9 mEq/L)	5955 (8.6)	476 (8.0)	2859 (8.6)
Prothrombin time > 14 s or PT international normalized ratio > 1.2	12,168 (17.6)	640 (5.3)	6364 (19.1)
Bands (>32%)	589 (0.8)	58 (9.8)	276 (0.8)
Platelets (115 × 10^9^/L)	2312 (3.3)	140 (6.1)	1164 (3.5)
Vital signs and altered mental status (AMS)			
Pulse (M49 or >129/min)	7051 (10.2)	529 (7.5)	3192 (9.6)
Pulse (120-129/min)	6459 (9.3)	274 (4.2)	2930 (8.8)
Pulse (100-119/min)	22.872 (33.0)	717 (3.1)	10.861 (32.6)
Oral temperature (<95 F)	826 (1.2)	75 (9.1)	300 (0.9)
Respirations (>39/min)	4101 (5.9)	297 (7.2)	1842 (5.5)
Respirations (30-39/min)	13,044 (18.8)	653 (5.0)	5818 (17.5)
Systolic blood pressure (£99 mm Hg)	6029 (8.7)	438 (7.3)	2887 (8.7)
Severe AMS	1728 (2.5)	344 (19.9)	770 (2.3)
Mild or moderate AMS	7044 (10.2)	538 (7.6)	3632 (10.9)
Major comorbiditics (sorted by prevalence)			
Hypertension	38.165 (55.1)	1151 (3.0)	19.462 (58.4)
Congestive heart failure	18.679 (27.0)	1080 (5.8)	9460 (28.4)
Diabetes without chronic complications	17,055 (24.6)	509 (3.0)	8762 (26.3)
Depression	10.158 (14.7)	264 (2.6)	5395 (16.2)
Deficiency anemias	10.032 (14.5)	531 (5.3)	5426 (16.3)
Peripheral vascular disease	5961 (8.6)	242 (4.1)	2917 (8.8)
Renal failure	4900 (7.1)	337 (6.9)	3603 (10.8)
Hematologic or solid organ malignancy	2410 (3.5)	136 (5.6)	1230 (3.7)
Diabetes with chronic complications	2379 (3.4)	107 (4.5)	1342 (4.0)
Pulmonary circulation disease	1950 (2.8)	246 (12.6)	1081 (3.2)
Weight loss	1816 (2.6)	203 (11.2)	997 (3.0)
Metastatic cancer	1028 (1.5)	93 (9.0)	527 (1.6)
Liver disease	896 (1.3)	37(4.1)	514 (1.5)

**Table 6:** Results from subgroups.

Subgroup	OR	*p* value	Weight
2000-2010	1.70 [0.97, 3.00]	0.07	21.7%
2011-2015	0.71 [0.56, 0.91]	0.007	44.2%
2016-present	1.12 [0.72, 1.73]	0.62	34.1%

## Data Availability

The data used in this study are available from the author upon request.
